# Tumor Region Location and Classification Based on Fuzzy Logic and Region Merging Image Segmentation Algorithm

**DOI:** 10.1155/2021/1141619

**Published:** 2021-10-20

**Authors:** Tianyu Zhao, Hang Dai

**Affiliations:** ^1^Medical Technology Department, Qiqihar Medical University, Qiqihar 161006, Heilongjiang, China; ^2^Foreign Language Department, Qiqihar Medical University, Qiqihar 161006, Heilongjiang, China

## Abstract

Early diagnosis of tumor plays an important role in the improvement of treatment and survival rate of patients. However, breast tumors are difficult to be diagnosed by invasive examination, so medical imaging has become the most intuitive auxiliary method for breast tumor diagnosis. Although there is no universal perfect method for image segmentation so far, the consensus on the general law of image segmentation has produced considerable research results and methods. In this context, this paper focuses on the breast tumor image segmentation method based on CNN and proposes an improved DCNN method combined with CRF. This method can obtain the information of multiscale and pixels better. The experimental results show that, compared with DCNN without these methods, the segmentation accuracy is significantly improved.

## 1. Introduction

The incidence of cancer has been rising worldwide in recent years. Because the cause of the disease is not clear, and treatment is difficult. Breast tumors, or tumors in breast tissue, can be divided into primary and metastatic according to their origin [1, 2]. In general, LGG has a benign tendency, well differentiated, and better prognosis, while HGG is a low differentiated and aggressive malignant tumor [3, 4]. Currently, the morbidity and mortality of breast tumors are increasing year by year.

Manual segmentation of breast tumor is a very tedious and boring work, and the segmentation of different operators, even the same operator at different times, is different. In addition, the boundaries of adjacent structures are often blurred due to the smooth intensity gradient, and the partial volume effect and partial field effect also increase the difficulty of segmentation [5, 6]. In recent years, many computer information processing technologies have been mature, and computers can help us handle a variety of information, but research shows that visual information accounts for more than 80% of the total human information, and traditional computer technology can only store and transmit such information and cannot handle such information. In order to use computer to deal with complex and rich visual information, digital image processing technology has been concerned and invested by people. Image processing technology is widely used in industrial production, medical image, security monitoring, image coding, satellite remote sensing, and other fields, so the research on digital image technology is a hot research topic in the field of computer science. Image segmentation is the process of dividing the image into different regions according to the content of the image. It is to separate the target region from the background which is not concerned, so as to improve the effectiveness of image description and classification.

There are many kinds of tumors. Starting from the research of breast tumors, the application of image segmentation algorithm based on fuzzy logic and regional merger in tumor classification, localization, and related algorithms is first introduced. Secondly, based on this technology, it carries out practical research on the classification and location of breast tumors and proposes a breast tumor image segmentation algorithm combining CRF and DCNN. The experimental results show that, compared with the classical breast tumor image segmentation technology based on CNN, this method can better obtain the multiscale and interpixel information and has certain advantages.

## 2. Related Concepts

### 2.1. Image Segmentation

The image in the sense of human vision is the result of imaging the reflected light of natural objects through the eyes, and the segmentation of human visual image is subjective and exists in the subconscious [1]. When an image is formed in human vision, human beings will segment the image into target area and background according to their own concerns or some characteristics of the image itself. However, using computer to process the digital image needs to judge how to segment the image through objective conditions. Therefore, we can use rigorous mathematical theory to describe the image segmentation.

The definition of image segmentation is expressed by the set theory in mathematics: the image domain *R* is represented by the set *t*, and the image segmentation of *R* is transformed into the nonempty subset *T*_*i*_ that *t* meets the following requirements:

1. ∪_*i*=1_^*n*^*T*_*i*_=*T*;
2. When *i* ≠ *j*, *T*_*i*_∩*T*_*j*_ = ∅;
3. When *i* is a natural number, *P* (*T*_*i*_) = true;
4. When *i* ≠ *j*, *PT*_*i*_∪*T*_*j*_=false;
5. When *i* is a natural number, *T*_*i*_ is connected;

Here, *p* (TI) is a logical predicate for all elements in the set *t*_*i*_.

Through these conditions, we can see the essence of image segmentation. The first point shows that all subregions of image segmentation are the original images. The second point shows that there are no same pixels between the subregions after segmentation, that is, one pixel exists and only exists in one region. The third and fourth points show that all pixels in a subregion have the same properties after segmentation, and there is no same property between pixels belonging to different subregions. The last point shows that any pixel in a region has connectivity.

### 2.2. Region Merging Algorithm

The region merging algorithm is to merge the small regions into larger regions according to the merging standard after the initial segmentation of the image and stop merging after reaching the stop standard. The effect of region merging algorithm is mainly affected by the merging standard. If the merging standard is not selected properly, the contour of the merged object will be lost.

Region adjacency graph can quickly find the adjacency relationship between two regions:

(1) $$\begin{array}{c} G=\left(V,E\right). \end{array}$$

In most cases, the gray mean value of the region in the image can represent the brightness characteristics of the image region. The smaller the difference of gray mean value between the two regions, the higher the similarity between the two regions should be. When other conditions are met, the two regions should be merged into a larger region. Therefore, the construction of regional gray difference evaluation function can reflect the similarity between different regions in the feature of brightness, which is one of the influencing factors of subsequent merging criteria. The traditional evaluation function of regional gray difference is as follows:

(2) $$\begin{array}{c} \delta R_{i},\;R_{j}=\frac{\left\|R_{i}\right\|\circ \left\|R_{j}\right\|}{\left\|R_{i}\right\|+\left\|R_{j}\right\|}{\left[\mu \left(R_{i}\right)-\mu \left(R_{j}\right)\right]}^{2}. \end{array}$$

In digital images, image regions have multidimensional attributes. In addition to the brightness attributes represented by gray values, they also include texture, boundary strength, and boundary geometric features. If the similarity between regions is judged only according to the gray difference of image regions, more important information will be lost in the final merging result. Therefore, we also need to select other attributes of the region to construct the difference evaluation function and gray difference value to form a composite regional similarity evaluation function in order to achieve better merging effect.

### 2.3. Fuzzy Algorithm

Fuzzy logic belongs to the theory of fuzzy mathematics, which is developed on the basis of fuzzy set theory. Through fuzzy logic, the computer can process fuzzy concepts in natural language.

In this paper, fuzzy logic system is used to calculate the merging degree of regions. Fuzzy logic system uses fuzzy sets and fuzzy rules to judge and reason. It can imitate human's judgment and reasoning thinking process of fuzzy concept, and can deal with fuzzy reasoning problems that traditional methods cannot deal with. At the same time, the regional merging system based on fuzzy logic system has the following advantages:

1. There is no need to build a mathematical model for the merging criteria. Fuzzy control is to build control rules according to human judgment process. It only needs to express human expert experience in natural language to quickly construct a fuzzy logic control system.
2. The fuzzy logic system has good robustness in dealing with both linear and nonlinear targets and has better adaptability than the traditional function method in dealing with nonlinear targets.
3. The calculation process of fuzzy logic system is composed of fuzzification, fuzzy reasoning, and defuzzification. As long as fuzzy semantics, fuzzy rule base, and membership function are input, a fuzzy logic system can be constructed, which is simpler than other methods.

The biggest difference between fuzzy set and classical set theory is that fuzzy set eliminates the nonzero or one discrete membership attribute of elements to class and makes the membership degree of elements to class continuous and linear. In classical set theory, the definition of set is as follows:

(3) $$\begin{array}{c} C_{A}\left(x\right)=\left\{\begin{array}{c} 1,\;x\in A,\\ 0,\;x\notin A. \end{array}\right. \end{array}$$

The definition of fuzzy set theory is as follows:

(4) $$\begin{array}{c} C_{A}\left(x\right)=\left\{\left(x_{i}⟶\mu_{A}\left(x_{i}\right)\right)\right\},\;x_{i}\in X. \end{array}$$

The formula of intermediate trapezoid function is as follows:

(5) $$\begin{array}{c} Ax=\left\{\begin{array}{c} x-a,\;a\leq x<b,\\ b-a,\;a\leq x<b,\\ 1,\;b\leq x<c,\\ d-x,\;c\leq x\leq d,\\ d-c,\;c\leq x\leq d,\\ 0,\;x<a\text{ or }d<x. \end{array}\right. \end{array}$$

The formula of intermediate Gaussian distribution function is as follows:

(6) $$\begin{array}{c} A\left(x\right)=e^{-{\left(\left(x-a\right)/\sigma \right)}^{2}},\;-\infty <x<+\infty . \end{array}$$

## 3. Tumor Location and Classification Method of Breast Tumor Image Segmentation

### 3.1. Database

In this paper, brats2015 is selected as the data source of the experiment. This is a breast tumor segmentation challenge initiated by the MICCAI conference in 2015 to evaluate and compare the latest methods in the current field [7, 8]. There are 220 HGG patients and 54 LGG patients in the public data brats2015. The images of each patient include four different imaging technologies: T1, T2, T1c, and flair. The training images are segmented into five labels: healthy breast tissue, necrosis, edema, and enhanced and nonenhanced tumor nuclei [9].

### 3.2. Cascade Structure

In this paper, the cascade structure, on the basis of ordinary cascade, enhances the division of labor before and after CNN and cascades different problems in turn. The first CNN is only responsible for segmenting the tumor from the background, and the segmentation result is used as the mask of the second CNN. The second (and subsequent) CNN is responsible for further dividing the tumor into specific substructures. In this test dataset, the tumor substructure is divided into four parts: necrosis, edema, enhanced tumor nucleus, and nonenhanced tumor nucleus. In order to simplify the subsequent segmentation task, we can cut out a small region from the global. In training, the region is generated from the standard data, while in testing, the region is generated from the result of the previous segmentation task [10, 11].

### 3.3. Evaluation Criteria

In this paper, the performance of the target method is quantitatively evaluated by three indicators, namely, dice similarity coefficient (DSC), sensitivity, and specificity (PPV). Their formula is as follows:

(7) $$\begin{array}{c} \text{DSC}=\frac{2\left|P\wedge T\right|}{\left|P\right|+\left|T\right|},\\ \text{sensitibity}=\frac{\left|P\wedge T\right|}{T},\\ \text{PPV}=\frac{\left|P\wedge T\right|}{P}, \end{array}$$

where *p* is the tumor region of the experimental segmentation result and *t* is the tumor region of the standard data.

## 4. Analysis of Test Results

### 4.1. Comparison of DSC, Specificity, and Sensitivity of Each Method

By comparing with other experimenters' methods, it can be found that our method is in the upper middle level in recent breast tumor image segmentation methods (Table 1). Firstly, methods based on DCNN are welcomed by researchers. More and more DCNN methods are used, and their segmentation results are obviously better than other methods. With the deepening of research, the advantages of other algorithms are absorbed and optimized continuously. Secondly, compared with other DCNN-based methods, this method has some advantages, which should be attributed to the use of ASPP structure and CRF. At the same time, the segmentation results of tumor nuclei, especially enhanced tumor nuclei, are more prominent, which has a great relationship with the application of cascade structure.

There are many reasons for the gap between this method and the best one. But the most important reason is that this method only convolutes in the two-dimensional plane, so it cannot synthesize the information of other pixels in the three-dimensional space. A simple method is to perform 2.5-dimensional convolution. The input information is no longer a single section, but a slice with thickness, which is inserted several times in DCNN.

Finally, we can synthesize the results of three different sections of the same point. The more complex but more valuable method is direct 3D convolution. The common 3D convolution has been quite mature. To expand ASPP to 3D, only 3D hole convolution is needed, and the theory and practice of CRF 3D are not difficult. Therefore, we can look forward to the improvement of this method.

Another huge limitation is that the training time of this method is large, so the number of iterations is less than other researchers, which affects the accuracy of segmentation results to a certain extent. At the same time, the experimental method is more complex than the control method, so the convergence speed may be slower under the same parameter setting. Therefore, after increasing the number of iterations, the advantages of the experimental method may be more obvious (Figure 1).

However, this is only an obstacle in the process of method research. In practice, there are good enough conditions and long enough training time. Therefore, this limitation does not seriously affects the feasibility of the method. After training, the method can quickly split test sets even on a PC, enough to meet practical needs (Figure 2).

### 4.2. Tumor Classification Test Results

According to Figure 3 and Table 2, the accuracy of tumor type discrimination is significantly higher than that of pathological analysis.

## 5. Conclusion

This paper proposes a breast tumor image segmentation method based on CRF and DCNN. In order to obtain multiscale information, a segmentation network structure is constructed by ASPP structure; in order to segment different levels of structure, segmentation is carried out step by step by cascade structure; in order to learn the relationship information between pixels, a CRF is added after DCNN. The experimental results show that, compared with DCNN breast tumor image segmentation technology without ASPP structure or CRF, the accuracy of this method is significantly improved. But compared with the latest 3D segmentation method, there is still a lot of room for improvement.

## Figures and Tables

**Figure 1:** PPV comparison of various methods.

**Figure 2:** Sensitivity comparison of various methods.

**Figure 3:** Accuracy of tumor classification based on this method.

**Table 1:** DSC comparison of various methods.

Method	DSC		
	Tumor whole	Tumor nucleus	Enhancement of tumor nucleus
CRF + integrated approaches	0.90	0.75	0.73
DeepMedic + CRF	0.90	0.75	0.72
InputCascade	0.88	0.79	0.73
DCNN	0.87	0.73	0.68
FCNN + CRF	0.85	0.73	0.62
Stacking denoising self-coding	0.82	0.68	0.64
SegNet	0.75	0.77	0.76
RF of pixel features	0.75	0.60	0.56

**Table 2:** Analysis of results.

	*n*	Calcification		Echo		Envelope		Morphological rules	
		Yes	No	Equality	Nonuniform	Yes	No	Yes	No
Optimum	39	7	32	28	11	34	5	33	6
Malignant	12	2	10	5	7	3	9	4	8

## Data Availability

The data underlying the results presented in the study are available within the article.
